The article "Blockchain Data Secure Transmission Method Based on Homomorphic Encryption" was published in 2022. Journal: Comput Intell Neurosci.

# Blockchain Data Secure Transmission Method Based on Homomorphic Encryption

**DOI:** 10.1155/2022/3406228

**Published:** 2022-04-30

**Authors:** Sheng Peng, Zhiming Cai, Wenjian Liu, Wennan Wang, Guang Li, Yutin Sun, Linkai Zhu

**Affiliations:** ^1^Faculty of Data Science, City University of Macau, Macau, China; ^2^Zhuhai Yingying Technology Co., Ltd, Zhuhai, China; ^3^Zhuhai College of Science and Technology, Zhuhai, China; ^4^Trusted Computing and Information Assurance Laboratory, Institute of Software Chinese Academy of Sciences, Beijing, China

## Abstract

To ensure the security of data transmission and recording in Internet environment monitoring systems, this paper proposes a study of a secure method of blockchain data transfer based on homomorphic encryption. Blockchain data transmission is realized through homomorphic encryption. Homomorphic encryption can not only encrypt the original data, but also ensure that the data result after decrypting the data is the same as the original data. The asymmetric encrypted public key is collected by Internet of things (IoT) equipment to realize the design of blockchain data secure transmission method based on homomorphic encryption. The experimental results show that the accuracy of the first transmission is as high as 88% when using the transmission method in this paper. After several experiments, the transmission accuracy is high by using the design method in this paper. In the last test, the transmission accuracy is still 88%, and the data transmission effect is relatively stable. At the same time, compared to the management method used in this article, the transfer method used in this paper is more reliable than the original transfer method and is not prone to data distortion. It can be seen that this method has high transmission accuracy and short transmission time, which effectively avoids the data tampering caused by too long time in the transmission process.

## 1. Introduction

Internet of things (IoT) has been evolving rapidly in recent years. The number of global Internet of things devices will increase by about 30% to 40% every year and will reach 20.8 million by 2020. In the fields of smart home, intelligent transportation, and industry, an IoT device is used to collect environmental information and send it to a centralized server for further processing or decision making. As more and more IoT devices appear in various versions, especially in critical systems, the need for secure data transfer between devices is increasing. At the same time, in order to realize the communication between numerous devices belonging to different organizations, Internet of things related solutions are seeking effective and reasonable methods and standards [1, 2]. At present, the problems faced by the centralized network architecture of the Internet of things are as follows:

1. If the centralized server fails, the whole network will be paralyzed. A Denial of Service (DOS) attack on a centralized server leads to a single point of failure.
2. Data stored in centralized servers lacks guaranteed accountability and traceability. The centralized system needs to trust a third party for data processing, and the stored data is at risk of deletion or tampering.
3. In the Internet of things, with the exponential growth of the number of Internet of things devices, the centralized server is not efficient in dealing with a large number of end-to-end communications. Therefore, the centralized approach may hinder the development of the Internet of things. Blockchain integrates and innovates with various technologies to protect data security, as shown in Figure 1.

In recent years, people pay more and more attention to blockchain technology. Blockchain is the core supporting technology represented by digital cryptocurrency [3, 4]. Blockchain technology has been applied to fields such as government, medical treatment, copyright, Internet of things, company management, Internet of vehicles, and so on and has promoted many business models that could not be realized previously. The so-called blockchain is a storage method for distributing data, which includes new data usage modes such as point-to-point data transfer, negotiation mechanisms, and encryption algorithms. It is a mode of data exchange by centralizing data and establishing corresponding database. During blockchain data transmission, data needs to be encrypted. Due to the old technology and easy decoding, the original encryption method often leads to the loss of data. Therefore, homomorphic encryption is used for data protection, which can detect and correct the data while encrypting to ensure the integrity of the data. Complete homomorphic encryption is a special method of encryption. Compared to the general homomorphic encryption algorithm, complete homomorphic encryption allows other people to receive encrypted data and perform any complex operation on the data without a decryption key. The whole process of computing can be entrusted to others. For example, the whole process of data encryption can not only reduce the cost of data access to others, but also transfer the whole process of computing to others. For example, the whole process of computing can be entrusted to others, which can reduce the cost of data encryption and so on. The data information on the blockchain is encrypted into ciphertext with homomorphic encryption algorithm. The smart contract on the blockchain can process ciphertext without knowing the plaintext information, which significantly improves the security of user data privacy [5, 6].

## 2. Related Works

In order to reach an agreement between decentralized blockchain nodes, all transaction logs in the blockchain must be disclosed to all nodes, which will greatly increase the risk of privacy breaches [7]. In the case of the use of cryptocurrency, analysts can analyze the transaction log to obtain the user's transaction style, as well as the user's personal information and location information [8]. We offer a reliable, personal OTT platform that handles the transaction process with a smart contract that is reliable and configurable. Smart contracts can be predefined for each product on a digital media content website (DMC) within the platform. After negotiating using a smart contract, a real data contract (RDC) is created and issued through a smart contract. A content producer or service provider can easily implement a trading strategy under a predefined smart contract [9]. In the industrial Internet of things (IIoT), energy transactions of decentralized nodes occur in various scenarios, such as microgrid, energy collection network, and vehicle to grid network. The alliance blockchain solves the common security and privacy problems caused by the untrusted and opaque energy market [10]. Huang J. and others proposed a new automatic food trading system based on alliance blockchain to improve trust and security in trading. It protects the privacy of stakeholders in the blockchain by using different authentication technologies [11]. Kumar S. S. and others realize the security and privacy protection of data sharing in electronic health system through alliance blockchain [12]. Thirukrishna. J. T. and others proposed CAIPY ecosystem based on smart contract to solve the cumbersome process problems in the field of insurance, which makes automobile insurance simple and transparent. CAIPY shows how smart contracts can support insurance companies without introducing new risks. Smart contracts have great potential to simplify these processes, thereby reducing costs [13]. Liu H. et al. adopted the smart contract technology based on Ethereum platform, established a hierarchical intelligent power distribution trading platform architecture for real-time transaction request and data acquisition, and realized the data security interaction under the high coupling of energy flow and information flow [14]. The combination of homomorphic encryption and Ethereum's smart contract technology makes it possible for insurance companies to obtain a customer's simple EHR text and claim object ID and decide whether to settle a claim even if patient information is not available, strengthening the confidentiality of any confidential information and user information disclosed to unauthorized users during interactions [15].

Based on this study, this paper suggests a reliable way to transfer data to a blockchain based on homomorphic encryption. In view of the problem of exposing data privacy in blockchain, taking user transactions as an example, this research is based on the fully homomorphic encryption algorithm without bootstrap conversion, combined with zero knowledge proof technology, under the account model, proposes the equal and full amount blockchain transaction protocol based on fully homomorphic encryption, and constructs a fully homomorphic encrypted data privacy blockchain based on intelligent contract. It can completely hide the input and output of the traditional blockchain trading system and the transaction details. Except for the transaction parties, the hidden details are completely invisible to anyone else. The threat that the transaction data information on the blockchain is analyzed by other malicious opponents will be greatly reduced, which significantly expands the application scenario of the blockchain.

## 3. Research Methods

### 3.1. Blockchain Related Technologies

#### 3.1.1. Block Structure

Blockchain consists of blocks containing transaction details. This information may be a transfer of cryptocurrency or other data exchange. Each block is logically divided into two parts: block header and block body. Each block is logically divided into two parts: the block head and the block body. Each block header contains the hash value of the previous block and other fields. Therefore, the blocks are connected in a similar way to the linked list as shown in Figure 2. Transaction information is stored in the block body. The first block in the blockchain is called the “genesis” block. The block hash value is obtained by a cryptographic hash, and each block stores the hash of the previous block, which helps keep the content in the blockchain unchanged. If hackers try to change the content of the previous blocks, the original hash value will be invalid. Hash values for subsequent blocks will be invalidated due to the domino effect. Therefore, if hackers want to change the content of a block, they must change the hash value in the header of all consecutive blocks and make corresponding changes in most nodes to reach a consensus [15, 16].

The transaction in the node verification block is part of the consensus algorithm [17]. Each transaction in the block has an ID value; this value is the hash value of the corresponding transaction information in the block. Make a hash of the transaction ID in pairs and create a hash tree inside the block body; see Figure 3. To sum up, the root of the hash tree is stored in the block header. Therefore, the Merkle tree branch containing the transaction can be used to perform verification without transaction verification through the local copy of the transaction. The tampered transaction will change the hash value in its branch, so that the tampered transaction can be detected without a lot of calculation.

#### 3.1.2. Consensus Algorithm

Consensus algorithm is an important part of blockchain. Its purpose is to safely update the system sharing state. In a blockchain system based on a “state machine copy,” the consensus algorithm ensures that the state of all copies remains synchronized and consistent at all times. The basic principles for developing a consensus algorithm are security, viability, and fault tolerance. Protection (n, f) refers to the degree of resistance to a system failure, such as a system that is resistant to force failure, where *n* is the total number of nodes, and *f* indicates the maximum number of nodes that the system can tolerate faults. The activity of consensus algorithm means that although there are *f* failed nodes, all correctly participating nodes can continue to reach distributed consensus. At any time, nodes may stop participating in consensus or take malicious actions. Consensus algorithm can be divided into two types: evidence-based consensus algorithm and voting based consensus algorithm. The following sections discuss examples of each type. In addition, the classification of various consensus algorithms is shown in Figure 4.

#### 3.1.3. Blockchain Type

Depending on how the blockchain is used in different applications, it can be divided into public blockchain, private blockchain, and consortium blockchain.  Table 1 lists detailed comparisons of three different blockchain types.

1. Public blockchain: public blockchain is a truly decentralized blockchain without any authority. Anyone is allowed to maintain the subsidiary wood of the blockchain and participate in the verification or release of new blocks. All members can access its content. In the public blockchain, publishing new blocks involves solving problems through a large number of calculations or holding their own cryptocurrency for a long time. As an incentive for the node to release the new block, each transaction in the block is accompanied by a transaction fee. This can encourage nodes to participate in consensus. At the same time, due to the higher cost of hackers tampering with the transaction content, it can effectively prevent the public blockchain from being attacked by hackers [18].
2. Private blockchain: Unlike public blockchain, each node in a private blockchain is a known member of an organization. A private blockchain is a database allocated by a single entity to control the exchange of information between different departments or individuals. It does not require cryptocurrency and does not charge a transaction fee.
3. Alliance blockchain: similar to the private blockchain, the alliance blockchain does not involve transaction costs, and the consensus calculation cost of publishing new blocks is not high. The difference is that the alliance blockchain spans multiple organizations. For auditable and reliable synchronized distributed databases, the alliance blockchain is used to track the data exchange between alliance members, which helps to ensure transparency among all parties.

### 3.2. Cryptography Related Technologies

#### 3.2.1. Hash Function

Hash function, a hash function called a hash algorithm, can create a fixed length hash value for any length of data. Hash values are usually represented by strings of random letters and numbers [19, 20]. All hash functions have the following basic properties: if the two hash values are different (according to the same hash function), the initial inputs of the two hash values are also different. This property has a descriptive property of the hash function. As a result, a hash function with this property is called a one-way hash function, as shown in Figure 5; if there is any character change in the input data, the output hash value will be very different, which is the input sensitivity of hash function. If you want to find two different strings and make their output hash values the same, it is not feasible to calculate in the strongly confused hash function, which reflects the anticollision of hash function.

#### 3.2.2. Asymmetric Encryption

The difference between asymmetric encryption and symmetric encryption is that it uses different keys in the process of encryption and decryption, which are called public key and private key, respectively. The public key and encryption algorithm can be made public, and the private key can only be kept by one party. When the receiving party decrypts the plaintext data using the plaintext private key, as shown in Figure 6, the receiving party encrypts the plaintext data using the plaintext private key. During digital signature, the sender uses its own private key to sign the message digest, and the receiver uses the sender's public key to verify whether the message digest comes from the sender. The process is shown in Figure 7.

### 3.3. Design of Blockchain Equivalent Transaction Protocol Based on Homomorphic Encryption

The blockchain equivalent transaction protocol based on homomorphic encryption uses zero knowledge proof technology to prove to miners that the ciphertext of the transaction amount encrypted by the transaction initiator with its own public key and the ciphertext of the transaction amount encrypted by the transaction receiver's public key contain the same plaintext information. When constructing a blockchain equivalent transaction protocol based on homomorphic encryption, if interactive zero knowledge proof is adopted, because there are many nodes in the blockchain, when the transaction initiator a (certifier) releases a transaction information, the miners on the blockchain need to interact with the transaction initiator A to verify the legitimacy of the transaction information. Because the interaction cost on the blockchain is very high, in a large blockchain network, miners will interact many times, which significantly affects the operation efficiency of the blockchain. Therefore, when constructing the blockchain equal value transaction protocol based on homomorphic encryption, this paper adopts noninteractive zero knowledge proof. The prover only needs to send a message to the verifier without interactive process, which is very important for blockchain [21, 22].

Suppose there is a transaction, the account balance of transaction initiator A is *t*_*A*_, and the transfer *t* amount needs to be sent to transaction receiver B.

The blockchain equivalent transaction protocol based on homomorphic encryption is described as follows:

Transaction initiator A encrypts the transaction amount *t* as *C*_*A*,*t*_ with its own public key, as shown in the following formula:

(1) $$\begin{array}{c} C_{A,t}\leftarrow \text{FHE}.\text{Enc}\left(pk_{A}.t\right). \end{array}$$

In (1), the random vector used for encryption is *r*_*A*,*t*_. Transaction initiator A encrypts *t* as *C*_*B*,*t*_ with the public key of transaction receiver B, as shown in the following formula:

(2) $$\begin{array}{c} C_{B,t}\leftarrow \text{FHE.Enc}\left(pk_{B}.t\right). \end{array}$$

In (2), the random vector used for encryption is *r*_*B*,*t*_. Transaction initiator A needs to prove the ciphertext *C*_*A*,*t*_ to the miner. The result of the computation of the plaintext information is equal to the result of the ciphertext information.

Input: security parameter *k* (hash length), ciphertext *C*_*A*,*t*_ of transaction amount *t* encrypted by A public key, and ciphertext *C*_*B*,*t*_ of *t* encrypted by A public key of B.

**Step 1 .**

A adds *C*_*A*,*t*_ and *C*_*B*,*t*_ into the empty zero knowledge proof bin.

**Step 2 .**

A generates a uniformly distributed random number *δ*_*i*_(1 ≤ *i* ≤ *k*).

**Step 3 .**

A calculates and generates the ciphertext of these K random numbers. A first encrypts the random number with its own public key, whose surname is *γ*_*A*,*i*_, as shown in the following formula:

(3) $$\begin{array}{c} \gamma_{A,i}\leftarrow \text{FHE.Enc}\left(pk_{A}.\delta_{i}\right). \end{array}$$

In formula (3), the random vector used for encryption is the weight *r*_*A*,*i*_, and then the public key of transaction receiver B is used to encrypt the random number *δ*_*i*_ as *γ*_*B*,*i*_, as shown in the following formula:

(4) $$\begin{array}{c} \gamma_{B,i}\leftarrow \text{FHE.Enc}\left(pk_{B}.\delta_{i}\right). \end{array}$$

In (4), the random vector used for encryption is *r*_*B*,*i*_. Finally, *γ*_*A*,*i*_ and *γ*_*B*,*i*_ are added to the zero knowledge proof *π*_1_′.

**Step 4 .**

A then calculates the sum of the ciphertext of the generated transaction amount *T* and the ciphertext of the random number *δ*_*i*_. A first performs homomorphic addition under its own public key, as shown in the following formula:

(5) $$\begin{array}{c} \Gamma_{A,i}=C_{A,t}+\gamma_{A,i}. \end{array}$$

Then the homomorphic addition operation is performed under the public key of transaction receiver B, as shown in the following formula:

(6) $$\begin{array}{c} \Gamma_{B,i}=C_{B,t}+\gamma_{B,i}. \end{array}$$

Finally, Γ_*A*,*i*_ and Γ_*B*,*i*_ are added to the zero knowledge proof *π*_1_′.

**Step 5 .**

A sends the zero knowledge proof *π*_1_′=(*C*_*A*,*t*_, *C*_*A*,*t*_, *γ*_*A*,*i*_, *γ*_*B*,*i*_, Γ_*A*,*i*_, Γ_*B*,*i*_) to the blockchain network.

**Step 6 .**

This section first considers constructing an interactive zero knowledge proof and then makes a slight change to turn the interactive zero knowledge proof into a noninteractive zero knowledge proof. The miner on the blockchain challenges a *h*, that is, the miner sends a string of *b*_*i*_ containing *k* bits to A (where *b*_*i*_ is evenly and randomly selected from {{0,1}).

**Step 7 .**

After receiving *h*, A gives different answers to miners according to different Bi. Specifically, if *b*_*i*_=0, A sends the plaintext information of *γ*_*A*,*i*_ and *γ*_*B*,*i*_ and the random vectors *r*_*A*,*i*_ and *r*_*B*,*i*_*i* required for encryption to the miners; if *b*_*i*_=1, A sends the plaintext information of Γ_*A*,*i*_ and Γ_*B*,*i*_ and the random vectors *r*_*A*,*i*_+*r*_*A*,*t*_ and *r*_*B*,*i*_+*r*_*B*,*t*_ required for encryption to the miners.

In general, the blockchain equivalent transaction protocol based on fully homomorphic encryption can verify whether the transaction amount reduced by account A is that the receiver wants A to publish the noninteractive zero knowledge proof 2 on the blockchain at one time. When publishing the transaction information, in order to increase the amount of account B, only A needs to publish the noninteractive zero knowledge proof *π*_1_ on the blockchain at one time [23].

### 3.4. Design of Blockchain Data Secure Transmission Method Based on Homomorphic Encryption

The basic framework of the blockchain data secure transmission method based on homomorphic encryption is shown in Figure 8 below.

The figure above shows the scope of a secure way to transfer blockchain data based on homomorphic encryption. The data transfer method completes the data transfer process by overlapping and computing, thus allowing the data to be transferred securely.

#### 3.4.1. Construction of Secure Transmission Block Unit Data Structure

From a macroperspective, the blockchain transmission method has designed a large number of algorithms and technologies. From a microperspective, blockchain refers to the data storage structure composed of microunits, which is used for the safe storage of some data to ensure that the data will not be tampered with at will. According to the corresponding characteristics of the blockchain and the hash pointer [3] data structure, the block structure is constructed [24, 25]. Some codes are as follows:

typedef struct block_ unit {

Char*∗* version.

unsigned int timestamp;

unsigned int height;

unsigned int term;

unsigned int trans num;

hash_ pt pre_ hash://Hash pointer.

mt hash root mkl root://MerkleRoot hash value.

mt_ t'mkl t; //pointMerklePointer to tree.

}block;

Through the above code writing, the block is constructed, and the part of the original block mode that does not adapt to homomorphic encryption is improved, so as to realize the structure suitable for the blockchain data secure transmission method based on homomorphic encryption.

#### 3.4.2. Homomorphic Encryption Calculation

The whole homomorphic encryption process is set as JK. It is known that the homomorphic encryption process consists of generating key, encrypting data, decrypting, and data evaluation. The generating key is set as kg, the encryption process is set as enc., the decryption process is set as Dec., and the evaluation process is eval. Then the formula can be expressed as

(7) $$\begin{array}{c} JK=\left(\text{KG,Enc,Dec,Eval}\right)\text{.} \end{array}$$

Suppose that the public key AK and the private key BK jointly generate the corresponding data security parameters, which are set to 0. AK is used to encrypt plaintext and BK is used to decrypt ciphertext. Set plaintext *Z* ∈ *Q*_*n*_, where *n* is an integer, and *Q*_*n*_ is a set of integers. The homomorphic encryption of *Z* is expressed as *W*_*c* *d*_(*c*), and the policy formula can be expressed as (8) and (9):

(8) $$\begin{array}{c} W_{c\;d}\left(v_{1}+v_{2}\right)=W_{cd}\left(v_{1}\right)⊕W_{c\;d}\left(v_{2}\right), \end{array}$$

(9) $$\begin{array}{c} W_{c\;d}\left(fv_{1}\right)=f⊗W_{c\;d}\left(v_{1}\right). \end{array}$$

The data is encrypted and transmitted through the above formula. At the same time, the data confidentiality process is carried out after the data is transmitted. Set the data decryption process to Dec. Decrypt ciphertext *e* through the private key, which can be expressed as the following formula:

(10) $$\begin{array}{c} u=\text{Dec}\left(E,AK\right). \end{array}$$

Finally, the decryption results are evaluated to complete the calculation process of homomorphic encryption. Assuming *L* is the evaluation function and the ciphertext is set to *e*, the evaluation algorithm evaluates the function *L* through the evaluation key *t*, so as to generate the evaluation ciphertext P. The specific formula is shown in the following formula:

(11) $$\begin{array}{c} P=\text{Eval}\left(T,i,E\right). \end{array}$$

The homomorphic encryption calculation process is completed through the above formula, and the calculation results are brought to the block structure in the above section through homomorphic encryption operation, so as to realize the safe transmission of data.

#### 3.4.3. Implementation of Blockchain Data Secure Transmission Method Based on Homomorphic Encryption

Through the above steps, the data is encrypted. In order to ensure the normal transmission process of the data, the IoT device is added to collect the data of the asymmetric encrypted public key in the data transmission process, set the obtained public key data as 129 bytes of encrypted data, and submit it to the nodes in the raft cluster through the homomorphic encryption path and save the public key data, decrypt it through the private key, and obtain the corresponding ID number [26]. Connect the data in the buffer area with the local blockchain to complete the data transmission.

## 4. Result Discussion

### 4.1. Comparative Analysis of Data Transmission Accuracy

The transmission results of this method and the transmission results of the original method are described in Figure 9. The specific results are as follows,

According to the comparative analysis of the data transmission accuracy in Figure 9, it can be seen that the data transfer method effectively improves the accuracy of the data transfer and reduces the distortion. To ensure the consistency of the results of this experiment, we performed a number of data transfer tests during the design period. As shown in Figure 9, when using the transmission method in this paper, the accuracy of the first transmission is as high as 88%. After several experiments, the transmission accuracy is high by using the design method in this paper. In the last test, the transmission accuracy is still 88%, and the data transmission effect is relatively stable. Comparing the management method used in this document with the original method, it can be seen that the transfer method used in this document is more reliable than the original method and is not as easy to distort the data.

### 4.2. Comparative Analysis of Data Transmission Time

In order to more intuitively reflect the advantages of this design method compared with the original data transmission method, the data transmission time is compared and described in detail through images, as shown in Figure 10.

As can be seen from Figure 10, the data transfer time of the information security blockchain based on the homomorphic encryption developed in this paper is relatively fast compared to the data transfer time of the original data transfer method. The first transfer method has a longer run time and less work efficiency. The transfer time of the original transfer method is unstable and it easily loses data. Therefore, the experience of using the first transmission method is poor. In this article, we can see that the blockchain information security method of transmission based on a kind of encryption has significantly improved the work efficiency and transmission accuracy.

## 5. Conclusion

In the future, the Internet of things will cover more areas of our daily life. This will lead researchers to pay more attention to the security problems of multidevice data transmission. Design a blockchain data secure transmission method based on homomorphic encryption. Blockchain data transmission is realized through homomorphic encryption. The hash pointer theory is used to encode, construct the data structure of secure transmission block unit, transmit data through homomorphic encryption, and use IoT equipment to collect the data of asymmetric encrypted public key, so as to realize the design of blockchain data secure transmission method based on homomorphic encryption. Build a comparison test; compared with the transmission method, this method has high transmission accuracy and short transmission time, which effectively avoids the data tampering caused by too long time in the transmission process. It can be seen that this method can better meet the actual transmission needs.

## Figures and Tables

**Figure 1:** Integration and innovation of blockchain and various technologies to protect data security.

**Figure 2:** Chain structure.

**Figure 3:** Block head and block body.

**Figure 4:** Consensus algorithm classification.

**Figure 5:** Hash encryption process.

**Figure 6:** Data encryption process.

**Figure 7:** Data signature process.

**Figure 8:** Blockchain data secure transmission method framework based on homomorphic encryption.

**Figure 9:** Comparison of transmission accuracy between this method and the original method.

**Figure 10:** Comparison of transmission time between this method and the original method.

**Table 1:** Comparison of different blockchain types.

	Public blockchain	Private blockchain	Alliance blockchain
Participating consensus members	All nodes	Single organization	Multiple organizations
Access control	Any member participates in reading/writing	Allow members to participate in read/write	Allow members to participate in read/write
Participant identity	Anonymous member	Licensed member	Licensed member
Invariance	Yes	Local	Local
Transaction processing speed	Slow	Fast	Fast
Decentralized trust	Slow	No	Local

## Data Availability

The data used to support the findings of this study are available from the corresponding author upon request.
